# Influences of Different Drop Height Training on Lower Extremity Kinematics and Stiffness during Repetitive Drop Jump

**DOI:** 10.1155/2021/5551199

**Published:** 2021-03-03

**Authors:** I-Lin Wang, Yi-Ming Chen, Ke-Ke Zhang, Yu-Ge Li, Yu Su, Chou Wu, Chun-Sheng Ho

**Affiliations:** ^1^College of Physical Education, Hubei Normal University, Huangshi 435002, China; ^2^Graduate Institute, Jilin Sport University, Changchun, 130022 Jilin, China; ^3^Division of Physical Medicine and Rehabilitation, Lo-Hsu Medical Foundation, Inc., Lotung Poh-Ai Hospital, Yilan 26546, Taiwan; ^4^Department of Physical Therapy, College of Medical and Health Science, Asia University, Taichung 41354, Taiwan

## Abstract

Drop jump (DJ) is often used as a plyometric exercise to improve jumping performance. Training from improper drop heights and for improper durations lead to unfavorable biomechanical changes in the lower extremities when landing, which result in reduced training effects and even lower extremity injuries. *Purpose*. To study the effects of repeated DJ training at drop heights of 30 cm, 40 cm, and 50 cm (drop jump height (DJH) 30, DJH40, and DJH50) on lower extremity kinematics and kinetics. The 1st, 50th, 100th, 150th, and 200th DJs (DJ1, DJs50, DJs100, DJs150, and DJs200) were recorded by using a BTS motion capture system and force platform. The MATLAB software was used to compare the kinematic and stiffness data of DJ1, DJs50, DJs100, DJs150, and DJs200 with one-way ANOVA repeated measure. If there were significant differences, the LSD method was used for post hoc comparisons. *Methods*. Twenty healthy male Division III athlete volunteers were selected as subjects, and 200 drop jumps (DJs200) were performed from DJH30, DJH40, and DJH50. *Results*. The jumping height (JH), contact time (CT), and GRF increased with drop height, and the stiffness of the legs and ankle at DJH30 was higher than that at DJH40 and DJH50 (*p* < 0.05). *Conclusion*. Within DJs200, training at DJH50 yield the high impact easily leads to lower extremity injury; training at DJH30 can increase the stiffnesses of the legs and ankle joints, thus effectively utilizing the SSC benefits to store and release elastic energy, reducing the risk of lower extremity musculoskeletal injury. Therefore, coaches can choose different drop heights and training quantities for each person to better prevent lower extremity injury.

## 1. Introduction

Plyometric exercise is a type of exercise in which the muscle is stretched directly before it is explosively contracted during the stretch-shortening cycle (SSC) to generate high levels of force and power, and the DJ is often performed during plyometric training [1]. DJ training with maximum vertical jumps performed immediately from a platform can be used to improve jumping performance [2]. Eccentric contraction during the downward phase immediately followed by a rapid concentric contraction during the takeoff is needed to complete DJ action with the participant of the SSC. However, an excessive landing force with decreased physiological absorption causes large knee valgus, which leads to lower extremity injury [3]. Therefore, too high of a drop height leads to excessive GRFs and lower extremity injury. The preactivation phase characteristics in DJ training systematically change with the drop height; therefore, lower extremity strength can be increased during DJ training [4]. Choosing the appropriate drop height during the DJ task can not only help improve performance by inducing the best training-related physiological adaptations but also help avoid injury to the muscle tendon and bone caused by overload on the lower extremities during jumps from high heights [5, 6]. Compared to the optimal drop height, a lower drop height results in interlimb asymmetry in strength [7], and a higher drop height does not enable small adjustments in muscle activity, which can even decrease rather than increase power output [4, 8]. Therefore, the optimal drop height may need to be selected according to the jumping ability of each participant [9].

In competitions, athletes jump and land multiple times to complete multiple high-intensity short-duration sprints, cuts, and spins [10], and all of these movements require a high level of reactive strength and force-generating capabilities of the lower extremities [11]. High athletic performance requires an adequate level of lower extremity strength [12], and DJ training yields adequate training effects [13]. Athletes usually perform plyometric jumps to improve their explosive jump performance, and the DJ is the most common plyometric exercise [6]. DJ training can improve muscle power by SSC mechanism, thereby enhancing athletic and vertical jumping performance [1, 14, 15]. Therefore, most athletes can use strength training with repeated jumps to improve the strength and biomechanical characteristics of the lower extremities. In addition, DJ training improves the ability of tendons and muscles to store and release elastic energy within the landing phase of jumps [16], thus increasing the lower extremity strength and allowing individuals to jump from higher heights. Jumping height can predict muscle strength in the lower extremities, so various vertical jumps are often included in a standard test of athletic performance [2]. However, repeated DJ training from different platforms is likely to lead to neuromuscular fatigue and changes in lower extremity dynamics, which can lead to injury. Landing strategies, including strategies of bouncing and absorbing energy, affect athletic performance [17], and improvements in the stretch reflex may lead to higher takeoff speeds [18]. The characteristics of preactivation can change with the drop height, and DJs from platforms higher than the optimal height do not allow the individual to effectively adjust muscle preactivation to adapt to the landing impact [4]; moreover, SSC fatigue after exercise leads to decreased stretch-reflex sensitivity and muscle injury during DJ training [19]. When repeated DJs performed with more extended lower extremities, the individuals induced muscle fatigue will increase ankle plantar flexion to absorb the impact forces as the compensation for increased knee extension and the change in landing strategy under this circumstance results in poor jumping performance [20]. A study showed that muscle performance changed after DJs100 was repeated, and knee joint extensor fatigue caused the jump height to decrease by 26 ± 14% [21]. Therefore, repeated DJ training is likely to induce lower extremity fatigue and muscle injury, and jumps from the optimal drop height and the optimal training volume for DJs can prevent the risk of poor performance and injury caused by excessive fatigue and help individuals complete reinforcement training.

The risk of lower extremity injury may be related to changes in joint stiffness; excessive joint stiffness increases the risk of bone injury, while insufficient joint stiffness may lead to joint instability and soft tissue injury [22]. DJ training from different drop heights is widely used to assess the risk of lower extremity injury [5], so drop height is a key factor affecting joint stiffness during landing. The optimal drop height can regulate the lower extremity stiffness, leading to the best SSC to enhance jumping performance [23]. Previous studies have shown that ankle stiffness decreases gradually with increasing drop height, resulting in smaller SSC benefits [6]. A drop height that is too high causes the DJ to overstretch the muscles during landing, decreasing lower extremity stiffness, which easily induces the neuroprotective inhibition process and reduces Hoffman reflex activity [24, 25]. An appropriate level of joint stiffness can effectively trigger the SSC mechanism to enhance the training effect, while repeated DJs induce muscle fatigue and changes in stiffness and the landing strategy, which limits jumping performance [20]. Therefore, the stiffness of lower extremity joints is affected by both drop height and training volume. The optimal drop height and training volume can effectively trigger the SSC mechanism to yield an appropriate stiffness, reduce the risk of lower extremity injury, and enhance jumping performance during repeated DJ training.

In summary, drop height and training volume affect DJ landing performance, and changes in these factors yield different training effects. An improper height and training volume lead to lower extremity musculoskeletal injuries. In this study, it was hypothesized that JH, CT, RSI, and GRF increase as the drop height and training volume increase and that stiffness decreases as the drop height increases. With the optimal drop height and training volume, the SSC mechanism may more effectively increase muscle spindle sensitivity, enhance endurance, improve athletic performance, and prevent lower extremity injury during DJ training. The main objectives of this study were to explore the training effects of highly repetitive DJs from DJH30, DJH40, and DJH50 on the kinematics and stiffness of the lower extremities.

## 2. Methods

### 2.1. Participants

The subjects involved in the study were 20 healthy male Division III athlete volunteers (age = 21.5 ± 0.9 years old, height = 174.6 ± 4.7 cm, weight = 67.9 ± 7.9 kg) from Jilin Sport University. None of the subjects had a history of muscle or bone issues in the lower extremity or neurological disease within 2 years. The procedure and possible risks were explained to subjects, and they signed written consent forms before the study began. The study was approved by the regional ethics committee, and all subjects signed informed consent forms (JLSU-IRB2020004).

### 2.2. Protocol

Before the study, the subjects performed a standard dynamic warm-up for the major muscle groups of the lower limbs (running on a treadmill at a speed of 8 km/h for 10 minutes). During the study, the subjects wore standard shoes provided by the laboratory to control for differences in the absorption characteristics of the soles of shoes. Three DJ experiments (DJH30, DJH40, DJH50) were conducted in a random order over 3 separate days, with 4 days of rest between each dropping height experiment. Before data collection, the subjects were required to practice the jump five times to ensure that their hands were on their waist and their feet were on the two force plates during the experiment. The subjects were encouraged to jump with maximum effort within the shortest ground contact time [26]. The data for DJ1, DJs50, DJs100, DJs150, and DJs200 were recorded, and a 10-second break was provided between jumps. The framework for the proposed methodology is shown in Figure 1.

### 2.3. Data Collection

Twenty-one reflective markers (19 mm in diameter) were attached to anatomical landmarks on the legs and pelvis to define a seven-segment rigid link model of the lower extremities, according to the Helen Hayes marker set [27]. The three-dimensional (3D) trajectories of the reflective markers on the participants were collected with 10 cameras (BTS DX400, BTS Bioengineering, Milano, Italy) at a sampling frequency of 200 Hz. Two force plates (40∗60 cm) were used to collect GRF data during each trial at a sampling frequency of 400 Hz (BTS P6000, BTS Bioengineering, Milano, Italy). The infrared camera data were synchronized with the force plate data via the Qualisys 64 channel A/D plate.

### 2.4. Data Analysis

A kinematic model was generated by defining the skeletal segments (foot, talus, shank, thigh of both extremities, and pelvis) in the standing trial. The central position of the hip joint was calculated by the method proposed by Bell et al. [28]. The center of the ankle joint was defined as the midpoint between the medial and lateral malleolus. The midpoint between the medial and lateral epicondyles was defined as the knee joint center. The anatomic coordinate systems of the thigh and shank were determined by the static calibration test. The vertical axis was defined as the line from the distal to proximal centers of the joint, while the anteroposterior axis was perpendicular to the vertical axis; the third axis was defined as the cross product of the anteroposterior and vertical axes and used to obtain the dynamic coordinate systems of the pelvis, thigh, and shank. We performed all calculations using a custom MATLAB program (Mathworks, Natick, RI, USA).

The landing phase was defined as the time interval from when the foot contacted the ground to the lowest center-of-mass position. A fourth-order low-pass Butterworth digital filter with a cutoff frequency of 50 Hz was used to smooth the GRF data. Jumping height (JH) was calculated by the following formula: JH = gT^2^/8. Contact time (CT) was defined as the time from initial ground contact to toe-off during the foot ground contact phase. The reaction strength index (RSI) was calculated as follows: RSI = JH/CT. The peak vertical ground reaction force (PVGRF) was defined as the maximum PVGRF at the initial point of contact with the ground to the maximum angle of knee flexion. The PGRF was normalized by the subjects' body weight (BW).

*K*_leg_ was calculated using the following formula:

(1) $$\begin{array}{c} K_{\text{leg}}\left(\text{BW}*\frac{\text{ht}}{\text{rad}}\right)=\frac{\text{vertical }{\text{GRF}}_{\text{hip}-\text{lowest}}}{{\Delta L}_{\text{leg}}}, \end{array}$$

where the vertical GRF at the lowest position of the hip joint is the vertical  GRF_hip−lowest_ and Δ*L*_leg_ represents the vertical displacement of the hip from the contact position to the lowest position [26].

*K*_joint_ was calculated by the following formula:

(2) $$\begin{array}{c} K_{\text{joint}}\left(\text{BW}*\frac{\text{ht}}{\text{rad}}\right)=\frac{{\Delta M}_{\text{joint}}}{{\Delta \theta }_{\text{joint}}}, \end{array}$$

where the change in joint moment between the instant of peak joint flexion and ground contact is defined as Δ*M*_joint_ and the angular displacement between the maximum joint flexion and the contact position is Δ*θ*_joint_.

### 2.5. Statistical Analysis

The MATLAB software (R2016a; MathWorks, Inc., Natick, MA) was used for various statistical analysis. The variables were analyzed using one-way ANOVA repeated measure for DJH30, DJH40 and DJH50 at DJ1, DJs50, DJs100, DJs150, and DJs200. When significant results were found, post hoc analysis was performed with LSD (*p* < 0.05) pairwise comparisons to compare the measured values between different drop heights. The effect size (ES) is used to determine whether a difference is a practical correlation difference. The modified Cohen scale was used to determine the size of variation differences in three drop height, <0.2 means trivial difference, 0.2-0.6 means small difference, 0.6-1.2 means moderate difference, and 1.2-2.0 means large difference [29].

## 3. Results

Figure 2 presents the mean deviations of each dependent kinematic variable of the lower extremities. Jumping height and contact time increased significantly overall (all *p* < 0.005) across the three increasing drop heights, and post hoc analysis revealed significant differences between DJH30, DJH40, and DJH50. Our results show that jumping height was 1.05-, 1.08-, 1.04-, 1.07-, and 1.08-fold higher (all *p* < 0.048; ES varying from 0.48 to 0.73) during DJH40 than DJH30; 1.13-, 1.15-, 1.07-, 1.13-, and 1.16-fold higher (all *p* < 0.006; ES varying from 0.71 to 1.35) during DJH50 than DJH30; and 1.07-, 1.07-, 1.04-, 1.06-, and 1.07-fold higher (all *p* < 0.046; ES varying from 0.48 to 0.67) during DJH50 than DJH40 at DJ1, DJs50, DJs100, DJs150, and DJs200, respectively (Figure 2(a)). The post hoc comparisons showed that contact time was 1.08-, 1.08-, 1.09-, 1.08-, and 1.07-fold higher (all *p* < 0.049; ES varying from 0.47 to 0.68) during DJH40 than DJH30; was 1.19-, 1.23-, 1.24-, 1.23-, and 1.18-fold higher (all *p* < 0.002; ES varying from 0.85 to 1.57) during DJH50 than DJH30; and 1.10-, 1.13-, 1.13-, 1.14-, and 1.11-fold higher (all *p* < 0.041; ES varying from 0.49 to 0.82) during DJH50 than DJH40 at DJ1, DJs50, DJs100, DJs150, and DJs200, respectively (Figure 2(b)). The reaction strength index value during DJH50 was significantly higher than DJH30 and DJH40 (*p* < 0.050), and the post hoc comparisons showed that during DJH50 was 1.14-fold (*p* = 0.048; ES = 0.47) higher than DJH30 and 1.14-fold (*p* = 0.021; ES = 0.56) higher than DJH40 at DJ1. The reaction strength index value during DJH40 was significantly higher than DJH30 and DJH50 (all *p* < 0.050), and the post hoc comparisons showed that the values were 1.08-, 1.06-, 1.12-, and 1.17-fold higher (all *p* < 0.028; ES varying from 0.54 to 0.74) during DJH40 than DJH30 and were 10.26%, 13.94%, 14.87%, and 13.14% lower during DJH50 than DJH40 (all *p* < 0.029; ES varying from 0.53 to 0.70) at DJs50, DJs100, DJs150, and DJs200, respectively (Figure 2(c)).

Figure 2 presents the mean deviations of each dependent ground reaction force variable for the lower extremities. The peak ground reaction force and leg ground reaction force significantly increased overall (all *p* < 0.050) across the three increasing drop heights, with the post hoc results showing differences between DJH30, DJH40, and DJH50. The post hoc comparisons showed that peak ground reaction force was 1.05-, 1.05-, and 1.07-fold higher (all *p* < 0.018; ES varying from 0.59 to 0.84) during DJH40 than DJH30 at DJs100, DJs150, and DJs200, respectively; 1.20-, 1.18-, 1.20-, 1.17-, and 1.21-fold higher (all *p* < 0.001; ES varying from 1.03 to 2.23) during DJH50 than DJH30; and 1.19-, 1.15-, 1.14-, 1.11-, and 1.13-fold higher (all *p* < 0.001; ES varying from 0.91 to 1.82) during DJH50 than DJH40 at DJ1, DJs50, DJs100, DJs150, and DJs200, respectively (Figure 2(e)). The post hoc comparisons showed that the right leg ground reaction force was 1.11-, 1.05-, and 1.06-fold higher (all *p* < 0.022; ES varying from 0.56 to 0.86) during DJH40 than DJH30 at DJs100, DJs150, and DJs200, respectively; 1.17-, 1.21-, 1.23-, 1.16-, and 1.18-fold higher (all *p* < 0.002; ES varying from 0.87 to 1.25) during DJH50 than DJH30; and 1.24-, 1.15 1.11-, 1.11-, and 1.11-fold higher (all *p* < 0.008; ES varying from 0.67 to 1.77) during DJH50 than DJH40 at DJ1, DJs50, DJs100, DJs150, and DJs200, respectively (Figure 2(d)). The post hoc comparisons showed that the left leg ground reaction force was 1.15-, 1.13-, 1.14-, 1.14-, and 1.15-fold higher (all *p* < 0.050; ES varying from 0.56 to 1.04) during DJH50 than DJH30 at DJ1, DJs50, DJs100, DJs150, and DJs200, respectively, and 1.08-, 1.10-, and 1.11-fold (all *p* < 0.005; ES varying from 0.72 to 0.81) higher than during DJH40 at DJs100, DJs150, and DJs200, respectively (Figure 2(f)).

Figure 3 presents the mean deviations of each dependent lower extremity stiffness variable. The leg and ankle stiffness decreased significantly overall (all *p* < 0.050) across the three increasing drop heights, with the post hoc results showing differences between DJH30, DJH40, and DJH50. The post hoc comparisons showed that the leg stiffness was lower during DJH40 than DJH30, with ∇ values of 10.46%, 15.43%, 17.62%, 12.38%, and 7.53% (all *p* < 0.047; ES varying from 0.48 to 0.64) and lower during DJH50 than DJH30, with ∇ values of 20.97%, 30.05%, 32.03%, 25.06%, and 23.82% (all *p* < 0.030; ES varying from 0.53 to 0.87) at DJ1, DJs50, DJs100, DJs150, and DJs200, respectively; the values were lower during DJH50 than DJH40, with ∇ values of 17.28%, 18.31%, 14.47%, and 17.62% (all *p* < 0.043; ES varying from 0.49 to 0.58) at DJs50, DJs100, DJs150, and DJs200, respectively (Figure 3(a)). The post hoc comparisons showed that ankle stiffness during DJH40 was lower than DJH30, with ∇ values of 19.35%, 32.00%, 25.00%, 19.30%, and 19.09% (all *p* < 0.040; ES varying from 0.18 to 0.91) and lower during DJH50 than DJH30, with ∇ values of 25.81%, 30.40%, 37.88%, 23.68%, and 30.00% (all *p* < 0.019; ES varying from 0.22 to 0.78) at DJ1, DJs50, DJs100, DJs150, and DJs200, respectively (Figure 3(d)). There were no significant differences in knee or hip stiffness between DJH30, DJH40, and DJH50 (Figures 3(b) and 3(c)).

## 4. Discussion

The purposes of this study were to investigate the effects of highly repetitive DJs from DJH30, DJH40, and DJH50 on lower extremity kinematics and stiffness and to determine the appropriate drop height and training volume of drop jump training. The results show that jumping height and contact time reached the maximum values within DJs200 at DJH50, and training at this height and volume can improve jumping performance; however, the large ground reaction force generates a high impact force, which can easily lead to lower extremity injury. Leg and ankle stiffness are maximal at DJH30, which can reduce the risk of lower extremity musculoskeletal injury and effectively utilize stretch-shortening cycle benefits to store and release elastic energy to improve jumping performance.

In this study, within DJs200, jumping height and contact time gradually increased with increasing drop height. Previous studies have shown that jumping height and contact time increase with increasing drop height [6, 30] and that the training intensity can be enhanced and the values of jump parameters such as jumping height and contact time can be influenced by the drop height [6]. However, some studies have shown that jumping height decreases with drop height [6]. Increased contact time results in increased knee flexion to absorb the increased landing force and thus greater jumping ability [7, 31]. And the long contact time with the ground can follow the natural trend of the substrate recoil, thus wasting a minimum amount of energy [32]. In this study, jumping height increased gradually with drop height, which may have been caused by the jumping ability increasing with increasing contact time. Therefore, the DJH50 height had a longer contact time than did different jumps and exhibited a jumping height increase, which may have produced a better training effect. In this study, reaction strength index was higher during DJH50 than during DJH30 and DJH40 at DJ1, while when landing, the reaction strength index was higher during DJH40, than during DJH30 and DJH50 at DJs50, DJs100, DJs150, and DJs200. The differences in reaction strength index according to the drop height and jump time are due to the changes in jumping height and contact time. The higher the jumping height and the shorter the contact time are, the higher the reaction strength index [33, 34]. Too high of a drop height altitude will produce a large landing impact and is not conducive to muscle fine-tuning which can even decrease rather than increase power output; after repeated DJs, muscle fatigue will lead to a smaller stretch-shortening cycle benefit and reaction strength index difference at different drop heights [4, 8, 19]. Thus, the gradual increase in drop height may lead to a change in the reaction strength index difference when the DJH40 and DJH50 jump times are different. This study showed that after DJ1, the DJH40 height produces a larger reaction strength index, which can have a larger training effect, while after repeat drop jump training at the DJH50 height, muscle fatigue may decrease the stretch-shortening cycle benefit, resulting in a decrease in the reaction strength index. Therefore, drop heights of DJH40 and DJH50 can produce greater reaction strength index values, and the reaction strength index value may be more suitable for drop jump training; however, training from DJH50 for 200 consecutive times produces a lower reaction strength index, which may easily cause muscle fatigue and poor jumping performance.

The results of this study show that the ground reaction force produced at DJH50 within DJs200 is greater than those produced at DJH30 and DJH40. Consistent with previous findings, our results show that the resistance training intensity can be controlled by the drop height, resulting in the ground reaction force gradually increasing with increasing drop height [35]. High drop heights cause individuals to land during DJs with high impact intensity [6], which can lead to ankle sprains, anterior cruciate ligament tears, and patellofemoral pain syndrome [36]. Therefore, landing with high impact during DJH50 can cause lower extremity injury and is not suitable for repeated contact time training. There were significant differences in ground reaction force between DJH30 and DJH40 at DJs100, DJs150, and DJs200. These differences may have been caused by the differences in the initial peak vertical ground reaction force at ground contact due to fatigue and individual changes in joint stiffness [17, 37]. Therefore, the impact force can be changed by controlling the training intensity at different drop heights. In this study, smaller ground reaction forces reduced the risk of lower extremity musculoskeletal injury when landing at DJ1, DJs50, DJs100, DJs150, and DJs200 from the height of DJH30.

In this study, during landing from DJH40 and DJH50 within DJs200, the stiffnesses of the legs and ankle joints were lower than those during landing from DJH30, while there were no differences in the stiffnesses of the knees and hips between other drop heights. Consistent with previous findings, the stiffnesses of the legs and ankle gradually decreased with increasing drop height, while the stiffnesses of the knees and hips did not significantly differ across drop heights [6, 26, 38]. The ankle stiffness decreased gradually with increasing drop height, resulting in a decrease in the stretch-shortening cycle benefit when drop jump training [6]; therefore, the smaller ankle stiffness may have affected the training effect. Increasing stiffness enables better storage and release of stretch-shortening cycle-based elastic energy [38]. In addition, jumping training can increase the joint stiffness of the lower extremities during landing, reduce the risk of injury, and improve athletic performance by strengthening the lower extremity muscles [39]. The higher leg and ankle stiffnesses generated by highly repetitive drop jump training at DJH30 in this study can lead to greater stretch-shortening cycle benefits regarding the storage and release of elastic energy and reduce the incidence of lower extremity injuries, which may be suitable for repetitive drop jump training. Past studies have shown that the longer the contact time at drop jump landing is, the lower the stiffness of the lower extremities [40]. In this study, contact time increased gradually with increasing drop height, so the stiffnesses of the legs and ankle may be related to the increase in contact time. Therefore, if athletes can consciously control the contact time during training, they may adjust the lower extremity stiffnesses at landing according to the drop height. The stiffnesses of lower extremity joints are affected by joint torques. In this study, the knee and hip stiffnesses showed no differences after repeated drop jump training, which may have occurred because the knee and hip torques did not change significantly between the drop heights. In summary, drop jump training with the appropriate lower extremity stiffness or stiffness adjustments during repeated jumping training can reduce the risk of lower extremity injury and enhance the training effect. This study showed that landing from the DJH30 height within DJs200 produces larger leg and ankle stiffnesses, which can yield greater stretch-shortening cycle benefits, thereby improving jumping performance and reducing the risk of lower extremity injury, so these parameters are suitable for repeated drop jump training.

### 4.1. Limitations

Limitations need to be considered when interpreting the results. Firstly, amounts of drop height are not sufficient, so we need lower and higher DJH such as 20 cm and 60 cm. Secondly, the subjects were obviously not blinded to the DJH, so the central nervous system may apply a protective strategy, and this could introduce performance bias. Thirdly, electromyographic was not used in this study, so the activity of the lower limb muscles is unknown during landing and jumping.

## 5. Conclusion

In summary, with increasing drop height, the kinematics and stiffnesses of the lower extremities varied during landing. DJ training from a high drop height produces a high impact intensity, resulting in a greater impact. Compared with the heights of DJH30 and DJH40, the DJH50 height yielded higher JH, CT, and GRF values, as well as smaller leg and ankle stiffnesses during landing; the changes in kinematics and stiffness by the drop height will affect the stability of the knee joint. Within DJs200, training at the height of DJH50 can yield better jumping performance; however, because the high impact easily leads to lower extremity injury, training at the drop height of DJH30 can increase the stiffnesses of the legs and ankle joints, thus effectively utilizing the SSC benefits to store and release elastic energy, improving jumping performance and reducing the risk of lower extremity musculoskeletal injury.

## Figures and Tables

**Figure 1:** Framework for the proposed methodology.

**Figure 2:** The jumping height, contact time, reaction strength index, the peak vertical GRF, and right and left leg GRF during drop jumps from three heights at DJ1, DJs50, DJs100, DJs150, and DJs200. Asterisk † indicates that a significant difference with DJH30; ‡ indicates that a significant difference with DJH40; § indicates that a significant difference with DJH50. *p* values <0.05 were considered to significantly differ.

**Figure 3:** The right leg, hip, knee, and ankle stiffness during drop jumps from three heights at DJ1, DJs50, DJs100, DJs150, and DJs200. Asterisk † indicates that a significant difference with DJH30; ‡ indicates that a significant difference with DJH40; § indicates that a significant difference with DJH50. *p* values <0.05 were considered to significantly differ.

## Data Availability

The data results are included in the manuscript.

## Abbreviations

DJ: Drop jump
DJH: Drop jump height
JH: Jumping height
CT: Contact time
SSC: Stretch-shortening cycle
RSI: Reaction strength index
BWs: Body weights
ES: Effective size
GRF: Ground reaction force
PGRF: Peak ground reaction force
RGRF: Right leg ground reaction force
LGRF: Left leg ground reaction force
PVGRF: Peak vertical ground reaction force.
